The article "Persistent Clostridium Difficile Diarrhea, Thinking Beyond Pseudomembranous Colitis: A Case Report" was published in 2021. Journal: Cureus.

# Persistent Clostridium Difficile Diarrhea, Thinking Beyond Pseudomembranous Colitis: A Case Report

**DOI:** 10.7759/cureus.20704

**Published:** 2021-12-26

**Authors:** Aeyidh K Alharbi, Mohammed Anjum Ahmed, Abdulhadi Tashkandi, Fahad A Alkhathaami, Abdulmalik I Alshehri

**Affiliations:** 1 Medicine, College of Medicine, King Saud Bin Abdulaziz University for Health Sciences, Riyadh, SAU; 2 Emergency Medicine, Prince Mohammed Bin Abdulaziz, Ministry of National Guard Health Affairs, Medina, SAU

**Keywords:** case report, pseudomembranous colitis, inflammatory markers, hemicolitis, c. difficile, bowel ischemia

## Abstract

The prevalence of *Clostridium difficile* infection (CDI) is increasing along with the availability of diagnostic tests and is becoming a common nosocomial infection. CDI is the cause of nearly all occurrences of pseudomembranous colitis as well as 10-25% of antibiotic-related diarrhea. In patients presenting with persistent *C. difficile* diarrhea, the most common cause is the recurrence of pseudomembranous colitis but other differential diagnoses may need to be considered. In this case, we report a case of *C. difficile* diarrhea associated with life-threatening colitis and bowel ischemia.

We report the case of a 60-year-old male with persistent *C. difficile* diarrhea complicated by bowel ischemia. He presented with one month of persistent diarrhea and vomiting that had been worsening over the past three days; these symptoms were precipitated with prolonged antibiotic use. The patient was not known to have any chronic diseases but was attending the oncology outpatient clinic for an undiagnosed colonic mass that needed further examination. The patient’s vitals showed tachycardia (116 bpm), and a palpable left lumbar mass was noted on examination. The patient’s laboratory tests revealed significantly high inflammatory markers and deranged renal functions, and x-ray images showed hemicolitis. The patient was admitted because of dehydration. Computed tomography (CT) of the abdomen was conducted which revealed bowel ischemia.

A high index of suspicion for bowel ischemia should be held in *C. difficile* cases presenting with persistent symptoms. *C. difficile* infection is a very common healthcare-associated infection, its risk factors are older age, hospitalizations, and severe diseases. There is a need to increase the awareness of clinicians and prompt the diagnosis if suspicion of complicated *C. difficile* is present such as bowel ischemia.

## Introduction

*Clostridium difficile* is a Gram-positive organism that was first discovered as the cause of antibacterial diarrhea and inflammation of the colon in the late 70s [1,2]. Mild diarrhea to hemodynamic crisis and death are some of the clinical manifestations. One of the most significant risk factors for the development of *C. difficile* colitis is recent antibiotic usage (less than two months); however, host and environmental factors also play a role [3,4]. *C. difficile* infection (CDI) is a very common healthcare-associated infection. The cardinal symptom is watery diarrhea, but it can present as other associated symptoms such as fever, abdominal pain, nausea, and vomiting. The main risk factor is antibiotic (e.g., metronidazole) use which may lead to disturbed microbiota in feces; additional risk factors are older age, hospitalizations, and severe diseases. The diagnosis is established by the presence of *C. difficile* toxin in stool and pseudomembranes observed on radiographic and colonoscopic evaluations [5].

The prevalence of CDI is increasing along with the availability of diagnostic tests and is becoming a common nosocomial infection. CDI is the cause of nearly all occurrences of pseudomembranous colitis as well as 10-25% of antibiotic-related diarrhea [6,7].

## Case presentation

A 60-year-old male patient presented to the emergency department of our hospital with a history of diarrhea and vomiting, which had worsened over three days. The patient had a similar history of one month of persistent diarrhea for which he had multiple healthcare visits and multiple antibiotics use (not documented ). On examination, he was dehydrated and exhibited tachycardia (116 bpm) but showed no other signs of hemodynamic instability. Abdominal examination revealed a palpable left lumbar mass, which was related to his undiagnosed colonic mass

The patient had also been attending an oncology outpatient clinic for an undiagnosed colonic and liver mass since the last two weeks of the above presentation, for which he was referred by a private clinic. He did not have any known chronic diseases.

In the emergency department, the patient underwent a further evaluation to determine the cause of his worsening symptoms. The patient’s laboratory tests revealed a raised C-reactive protein (CRP) level of 247 mg/L (normal range: 0.1-4.9 mg/L), leukocytosis of 45,000 WBCs per microliter (normal range: 4500-11,000 WBCs per microliter), blood urea nitrogen of 11 mmol (normal range: 2.1-8.5 mmol), and a raised lactic acid level of 4.23 mmol/L (normal: less than 2.2 mmol/L) (Table 1).

**Table 1:** Laboratory value WBCs: white blood cells

Lab test	First day	Second day	Normal range
C-reactive protein (CRP)	247 mg/L	313 mg/L	0.1-4.9 mg/L
Leukocytosis	45,000 WBCs per microliter	24100 WBCs per microliter	4500-11,000 WBCs per microliter
Blood urea nitrogen	11 mmol	13.6 mmol	2.1-8.5 mmol
Lactic acid level	4.23 mmol/L	2.34 mmol/L	Less than 2.2 mmol/L

Abdominal x-ray revealed prominent air-filled bowel loops in the small and large intestines and mucosal thickening with luminal narrowing of descending colon indicating left hemicolitis (Figure 1). The patient showed signs of improvements after adequate hydration, with lactic acid decreasing to 2.34 mmol/L. His stool analysis tested positive for *C. difficile*. Accordingly, the patient was discharged home on oral vancomycin and metronidazole medication.

**Figure 1:** Abdominal x-ray showing mucosal wall thickening with narrowing in the lumen of the descending colon (yellow arrows).

However, the patient came back to the emergency department the next day with worsening diarrhea and vomiting. The repeat abdominal examination showed the same findings as to the previous one. However, his laboratory tests revealed increased blood urea nitrogen (BUN) (13.6mmol), increased CRP (313 mg/L), and lactic acid (2.43 mmol/L) levels.

Abdominal computed tomography (CT) revealed acute and chronic portal, superior, and inferior mesenteric thrombosis and thrombosis in the left side tributaries and splenic veins with subsequent bowel ischemia in the jejunum and left colon evident by decreased mural enhancement with mural thickening and luminal narrowing of the descending colon, without evidence of malignancy in the chest, abdomen, and pelvis (Figures 2-5).

**Figure 2:** Abdominal computed tomography with contrast (coronal view) showing decreased mural enhancement with mural thickening and luminal narrowing of the descending colon (yellow arrows).

**Figure 3:** Computed tomography, sagittal view, showing decreased mural enhancement with mural thickening and luminal narrowing of the descending colon (yellow arrows).

**Figure 4:** Computed tomography showing mural thickening at the hepatic flexure (blue arrow) and splenic flexure (yellow arrow).

**Figure 5:** Computed tomography showing sigmoid colon mural thickening and luminal narrowing with decreased enhancement (yellow arrows).

The patient was subsequently managed conservatively (isolation, low-molecular-weight heparin, nil per os, parenteral nutrition, and antibiotic regimen of metronidazole and vancomycin). No surgical intervention was recommended. His symptoms improved, and he was discharged after seven days. On follow-up of the patient in the outpatient department after two weeks, all his symptoms had improved. Interestingly, the undiagnosed colonic mass also regressed in the physical examination following the treatment for the ischemia, indicating that this mass might have only been secondary to bowel ischemia.

## Discussion

The majority of cases can be treated with antibiotics such as metronidazole or vancomycin to impede *C. difficile* overgrowth and toxin generation in the colon; however, there is a wide range of diseases; in some patients, life-threatening systemic toxicity occurs despite proper and rapid medical treatment [8,9]. Instead of bacteremia, colonic perforation, or ischemia, pathogen inflammatory response (interleukin-8, macrophage-inflammatory protein-2, substance P, and tumor necrosis factor) causes systemic consequences [10,11]. A patient with the first recurrence has a higher risk of subsequent recurrence and may start a cycle of several episodes, which can lead to tiredness and extended antimicrobial treatment courses. Apart from *C. difficile* infection, asymptomatic colonization (the presence of the bacteria without signs of *C. difficile* infection) occurs in 4-15% of healthy people [12]. A recent study found that asymptomatic colonization by a toxigenic strain during hospital admission increased the probability of CDI later [13]. Furthermore, asymptomatic *C. difficile* carriers shed the bacteria into the environment, and a growing body of evidence suggests that asymptomatic carriers play a key role in establishing and maintaining transmission in the ward [13]. It is unclear why some patients experience more severe symptoms than others, but it could be associated with the host’s ability to build an effective antibody-mediated response to clostridial toxins [14,15]. Unknown geographic factors appear to play a significant effect in the occurrence and severity of the disease.

In hospitalized patients, the incidence of *C. difficile* colitis increased from 0.68% to 1.2% in 2000, and the incidence of *C. difficile* colitis in patients who had life-threatening symptoms increased from 1.6% to 3.2% [16]. Risk factors included a previous surgical operation and immunosuppression. *C. difficile* colitis was 46 times more common in lung transplant patients, and severe illness was eight times more common. All patients were correctly diagnosed using an abdominal CT scan, but 12.5% of toxin tests and 10% of endoscopies were erroneously negative. The total mortality rate for patients receiving colectomy for *C. difficile* colitis was 57%. Preoperative vasopressor needs and age were both significant predictors of mortality after colectomy [16].

It was observed that if development to a more fulminant course was caused by a combination of an infectious and an ischemic event in some of the more severe patients with the probable scenario that severe diarrhea caused by *C. difficile* causes dehydration and a relative decrease in blood pressure, leading to either global or localized intestinal ischemia, which accelerates the likelihood of developing a systemic inflammatory response syndrome and having a more acute presentation. The notion that the opposite happens - that earlier relative intestinal ischemia causes greater sensitivity to the toxin and a more severe presentation - is fascinating, especially considering the findings of the study by Dallal et al. [16,17].

Colonic wall thickening and colon wall nodularity are two contrast-enhanced computed tomography (CECT) findings that reflect *C. difficile* infection (CDI) in the intestine. With the exception of Crohn's disease, the most prevalent finding in *C. difficile* infection is colonic wall thickening, which can be circumferential or eccentric and is typically more evident in comparison to other inflammatory colonic illnesses [18]. CDI can damage isolated sections of the colon or rectum, despite its rarity [18]. There have been a few occurrences of small bowel involvement documented in the literature, mostly as isolated case reports, especially in individuals with surgically changed small intestinal architecture [19,20].

## Conclusions

The current patient had multiple healthcare visits and multiple antibiotic uses for one month due to persistent diarrhea and vomiting, with undiagnosed colonic mass. Presented to the ER with worsened symptoms over the course of three days, his stool analysis tested positive for *C. difficile*. After the initial treatment symptoms improved and discharged, then suddenly a day after, he came back to the ER with a severe condition, CT revealed subsequent bowel ischemia. The patient was managed conservatively, his symptoms improved, and he was discharged after seven days. On follow-up of the patient after two weeks, all his symptoms had improved. Interestingly, the colonic mass also regressed. Finally, a high index of suspicion for bowel ischemia should be held in *C. difficile* cases presenting with persistent symptoms.
